The article "Generalized linear modeling of HCV infection among medical waste handlers in Sidama region, Ethiopia" was published in 2025. Journal: Front Epidemiol.

# Generalized linear modeling of HCV infection among medical waste handlers in Sidama region, Ethiopia

**DOI:** 10.3389/fepid.2024.1485482

**Published:** 2025-01-06

**Authors:** Birhanu Betela Warssamo

**Affiliations:** Department of Statistics, College of Natural and Computational Science, Hawassa University, Hawassa, Ethiopia

**Keywords:** hepatitis C virus, risk factors, waste handlers, prevalence, Sidama Ethiopia

## Abstract

**Background:**

There is limited evidence on prevalence and risk factors for hepatitis C virus (HCV) infection among waste handlers in Sidama region, Ethiopia; however, this knowledge is necessary for effective prevention of HCV infection in the region.

**Methods:**

A cross-sectional study was conducted among randomly selected waste collectors from October 2021 to 30 July 2022 in different public hospitals of Sidama region of Ethiopia. Serum samples were collected from participants and screened for anti-HCV using rapid immunochromatography assay. Socio-demographic and risk factor information of waste handlers was gathered by pretested and well-structured questionnaires The generalized linear model (GLM) was conducted using R software, and *P*-value <0.05 was declared statistically significant.

**Results:**

From a total of 282 participating waste handlers, 16 (5.7%) (95% CI = 4.2–8.7) were infected with hepatitis C virus. Educational status of waste handlers was the significant demographic variable that was associated with hepatitis C virus (AOR = 0.055; 95% CI = 0.012–0.248; *P* = 0.000). More married waste handlers, 12 (75%), were HCV positive than unmarried, 4 (25%) and married waste handlers were 2.051 times (OR = 2.051, 95% CI = 0.644–6.527, *P* = 0.295) more prone to HCV infection, compared to unmarried, which was statistically insignificant. The GLM showed that exposure to blood (OR = 8.26; 95% CI = 1.878–10.925; *P* = 0.037), multiple sexual partners (AOR = 3.63; 95% CI = 2.751–5.808; *P* = 0.001), sharp injury (AOR = 2.77; 95% CI = 2.327–3.173; *P* = 0.036), not using personal protective equipment (AOR = 0.77; 95% CI = 0.032–0.937; *P* = 0.001), contact with jaundiced patient (AOR = 3.65; 95% CI = 1.093–4.368; *P* = 0.0048) and unprotected sex (AOR = 11.91; 95% CI = 5.847–16.854; *P* = 0.001) remained statistically significantly associated with HCV positivity.

**Conclusions:**

The study revealed that there was a high prevalence of hepatitis C virus infection among waste handlers in Sidama region, Ethiopia. This demonstrated that there is an urgent need to increase preventative efforts and strategic policy orientations to control the spread of the hepatitis C virus.

## Introduction

Inflammation of the liver caused by hepatitis C virus (HCV) is hepatitis C infection. Acute and chronic forms of hepatitis C, ranging from mild sickness to severe, long-term infections including liver cirrhosis and cancer, are caused by this virus (1). The primary modes of exposure and transmission of HCV among medical waste handlers are associated with blood-to-blood contact through unsafe waste management practices. It can be transmitted via prenatal infection, skin and mucous membrane infections caused by contaminated blood or body fluid, sexual contact, and injection drug abuse. Additionally, skin art, ear/nose piercing, sharp injuries, and abortion can be the cause of infection. Hepatitis C is not transmitted via maternal milk, food, water, or casual contact such as hugging, kissing, and sharing food or drink with an infected individual (2).

The article "Generalized linear modeling of HCV infection among medical waste handlers in Sidama region, Ethiopia" was published in 2025. Journal: Front Epidemiol.

As of the most recent data from 2024, approximately 1.3 million people died from viral hepatitis in 2022, an increase from 1.1 million in 2019. Of these deaths, around 221,000 people died from hepatitis C in 2022. This is part of an ongoing global issue where hepatitis C is leading causes of liver-related deaths. Despite improved treatments and diagnostics, access to care remains limited in many regions, and global death rates have risen (3).

Hepatitis C virus is a world health problem. In occupational situations, waste handlers are exposed to hazardous blood-borne pathogens (an organism causing disease to its host) such as HCV. The problems of HCV have been the seventh primary cause of death globally. Viral hepatitis causes approximately 1.4 million deaths each year (4). HCV is a common cause of work-related infections passed from patients to waste handlers and the reverse and also to waste handlers' families. HCV infections can also be a cause for psychological and occupational diseases (5).

WHO estimation showed in 2017 that 58 million people globally were living with hepatitis C, 1.5 million people were newly infected with chronic form hepatitis C and it is the source of liver cancer and cirrhosis (6). HCV occurs in all regions including Eastern Mediterranean Region and European Region, with an estimated 12 million people chronically infected in each region. In African Region 9 million people are chronically infected, and 5 million people are infected in Region of the Americas. The prevalence of anti-HCV in Ethiopia ranged from 0% to 22% (7).

Infection with HCV does not permanently need treatment since the immune system in some individuals will clear the infection. But, when the infection becomes chronic, treatment is needed. WHO recommends therapy with pan-genotypic direct-acting antivirals (DAAs), for those adults and children with age below 3 years and with a chronic form of hepatitis C infection, but this therapy may remain costly especially in low-income countries like Ethiopia. Thus, WHO recommends prevention using personal protective equipment and infection prevention measures.

The article "Generalized linear modeling of HCV infection among medical waste handlers in Sidama region, Ethiopia" was published in 2025. Journal: Front Epidemiol.

In Ethiopia, data on the transmission of infection due to waste handling is scarce, and work-related exposure to waste may cause HCV infection (8). For effective prevention, sufficient information on the prevalence and associated risk factors of HCV is necessary. No studies have been conducted on HCV infection and risk factors among waste handlers in Sidama region, Ethiopia. Furthermore, people infected with HCV can develop symptoms between two weeks and six months later, and they may unknowingly infect others. Early detection and treatment can help prevent serious liver damage and infection progression. Hence, this study was aimed to determine HCV infection and risk factors among waste handlers in Sidama region, Ethiopia.

## Methods and materials

### Study design and setting

A cross-sectional study was used in four different governmental hospitals such as Hawassa University Comprehensive Specialized Hospital, Yirgalem General Hospital, Aleta Wondo Primary Hospital and Bensa Daye General Hospital found in Sidama National and Regional State (SNRS), Ethiopia, from October 2021 to July 30, 2022.

### Sampling procedures

A multistage sampling technique was adopted, and the facilities were then divided into hospitals. A lottery method was used to select four hospitals from a total of eighteen hospitals in Sidama region, Ethiopia.

### Data gathering and quality control

The questionnaire was written in English, translated back into the local language (Amharic and Sidamigna), and then translated back into English to ensure consistency. It was pre-tested on 10% of the sample size working at hospitals that were not included in the study to ensure validity and completeness. The data collectors were constantly monitored to ensure the reliability of the data. After obtaining informed written consent from each participant, the data were collected on socio-demographic characteristics and occupational and non-occupational risk factors for hepatitis C virus exposure using a pretested structured questionnaire. A random selection method was used in each hospital to select study participants who were employed by healthcare facilities and in good health condition to be able to answer questions. Those waste collectors who did not participate in or were exposed to waste management, were mentally ill, or seriously ill, and had a history of HCV infection prior to employment were excluded. In data gathering, the information was checked for completeness every day by supervisors and investigators after it was collected.

The article "Generalized linear modeling of HCV infection among medical waste handlers in Sidama region, Ethiopia" was published in 2025. Journal: Front Epidemiol.

### Laboratory testing

About 5 ml of venous blood was collected from all study participants according to the standard blood collection procedure. Separated sera were transported to the laboratories of Hawassa University Comprehensive Specialized Hospital and Yirgalem General Hospital using a cold box and stored at—20°C until tested. All serum samples from waste handlers were screened for anti-HCV using rapid immunochromatography assay. All tests were performed according to the manufacturer's instructions and samples positive for HCV sero-markers were rechecked by the same method.

### Study subjects

The study subjects were waste handlers from different public hospitals in Sidama National and Regional State. By lottery method we selected four hospitals from the region and there were total of 1,116 waste handlers in four hospitals (340 in Hawassa University Comprehensive Specialized Hospital, 258 in Yirgalem General Hospital, 234 in Aleta Wondo Primary Hospital and 284 in Bensa Daye General Hospital. Involvement in the study was on a willing basis, and all participants gave informed written consent.

### Sample size determination

The appropriate sample size used for this study was obtained using the following formula (9).

$$n=\frac{Z^{2}P(1-P)N}{d^{2}(N-1)+Z^{2}P(1-P)}$$

where *n* is the required total sample size, *N* is the total number of waste handlers in the study region, *Z* is the standard normal cumulative distribution that corresponds to the 5% level of confidence (*Z* = 1.96), *d* is the level of precision (sampling error), and *P* is the prevalence of HCV among waste handlers which is determined from previous studies which is 0.2. The level of precision preferred for this study was 4%. The desired sample size from the target population was 282 study subjects. The sample size was distributed into four hospitals using proportional allocation, $n_{h}=(N_{h}/N)*n$, where $n_{h}$ is the sample size for stratum *h*, $N_{h}$ is the population size for stratum *h*, *N* is the total population size and *n* is total sample size. Using the proportional allocation, 86 waste handlers were selected from total waste handlers working in Hawassa University Comprehensive Specialized Hospital, 66 from total waste handlers working in Yirgalem General Hospital, 59 from total waste handlers working in Aleta Wondo Primary Hospital and 71 from total waste handlers working in Bensa Daye General Hospital.

### Data processing and analysis

The collected data was entered into SPSS version 20 statistical package for data cleaning and the *n* exported to R software for analysis. Descriptive summary measures were calculated using a frequency table, percentages, and mean and standard deviation. The risk of association was assessed using the chi-square test. Variables having *P*-values less than 0.05 in the bivariate analysis were included in the multivariate analysis. Generalized linear regression analysis was employed at a 95% confidence interval to determine the presence of an association between risk factors and HCV infection. *P*-value <0.05 at 95% CI was taken as statistically significant.

The article "Generalized linear modeling of HCV infection among medical waste handlers in Sidama region, Ethiopia" was published in 2025. Journal: Front Epidemiol.

## Results

### Socio-demographic characteristics of waste handlers

Blood samples were collected and 282 waste handlers were involved in the study. Data on socio-demographic characteristics had already been reported in the published paper (10) and data on risk factors for HCV were obtained from all study participants. The mean age of the respondents was 37.13 years with a standard deviation of 14.42 and range of 18–65 years.

Socio-demographic characteristics of waste handlers and their association with HCV infection are shown in Table 1. As indicated, not statistically significant associations of HCV infection were detected in age (OR = 0.245; 95% CI = 0.042–6.742; *P* = 0.172), gender (OR = 1.41; 95% CI = 0.125–2.349; *P* = 0.132), marital status (OR = 2.051, 95% CI = 0.644–6.527; *P* = 0.295), accommodation (OR = 0.396; 95% CI = 0.12–1.303; *P* = 0.122), total family size (OR = 1.778; 95% CI = 0.281–2.150; *P* = 0.798), residence (OR = 2.833; 95% CI = 0.856–9.383), and years of experience (OR = 1.667; 95% CI = 0.236–1.887; *P* = 0.607) among waste handlers, and a significant association was identified in educational level (OR = 0.055; 95% CI = 0.012–0.248; *P* = 0.001).

**Table 1:** Socio-demographic characteristics of waste handlers and their association with HCV infection (*n* = 282).

Variables	Categories	Anti-HCV status		OR (95% CI)	*P*-value
		Positive *n* (%)	Negative *n* (%)		
Age	≥37	11 (68.8)	123 (46.2)	1	0.172
	<37	5 (31.2)	143 (53.8)	0.245 (0.042–6.742)	
Gender	Male	4 (25)	32 (12)	1	0.132
	Female	12 (75)	234 (88)	1.41 (0.125–2.349)	
Educational level	Elementary and below	14 (87.5)	74 (27.8)	1	0.001*
	Secondary and above	2 (12.5)	192 (72.2)	0.055 (0.012–0.248)	
Marital status	Single	4 (25)	108 (40.6)	1	0.295
	Married	12 (75)	158 (59.4)	2.051 (0.644–6.527)	
Accommodation	Living alone	4 (25)	31 (11.7)	1	0.122
	Not alone	12 (75)	235 (88.3)	0.396 (0.12–1.303)	
Total family size	<5	9 (56.2)	133 (50)	1	0.798
	≥5	7 (43.8)	133 (50)	1.778 (0.281–2.150)	
Residence	Urban	12 (75)	238 (89.5)	1	0.093
	Rural	4 (25)	28 (10.5)	2.833 (0.856–9.383)	
Years of experience	≥8	10 (62.5)	140 (52.6)	1	0.607
	<8	6 (37.5)	126 (47.4)	1.667 (0.236–1.887)	

* Significant variable.

The article "Generalized linear modeling of HCV infection among medical waste handlers in Sidama region, Ethiopia" was published in 2025. Journal: Front Epidemiol.

More married waste handlers, 12 (75%), were HCV positive than unmarried 4 (25%), and married waste handlers were 2.051 times (OR = 2.051, 95% CI = 0.644–6.527, *P* = 0.295) more prone to HCV infection, compared to unmarried. The prevalence of HCV infection was higher among females 12 (75%) than males 4 (25%) and more urban dwellers, 12 (75%), were HCV positive compared to rural 4 (25%). Odds of having HCV infection were 0.055 times less common among waste handlers who were secondary and above in their educational status (OR = 0.055, 95% CI = 0.012–0.248, *P* = 0.000), compared to waste handlers with elementary and below level of education and odds of acquiring HCV infection were 1.667 times more common among waste handlers who had greater than 8 years' experience of cleaning wastes (OR = 1.667, 95%CI = 0.236–1.887, *P* = 0.607), compared to waste handlers who cleaned wastes for 8 and less years of service. Waste handlers who had family size greater than or equals to five were 1.778 times more likely to acquire HCV infection (OR = 1.778, 95% CI = 0.281–2.150, *P* = 0.798), compared to those who have family size of less than five (Table 1).

### Prevalence of hepatitis C infection among study subjects

According to the finding of this research, 16 (5.7%) (95% CI = 4.2–8.7) of the respondents tested positive for anti-HCV (Table 2).

**Table 2:** Prevalence of HCV among waste handlers in public hospitals in Sidama region, Ethiopia, 2022 (*n* = 282).

Variable	Status	Number (%)
Anti-HCV antibody	Positive	16 (5.7)
	Negative	266 (94.3)

There were a statistically significant difference in the rate of HCV infection among study participants' risk factors (*P* > 0.05), with the exception of body/gum tattooing. Among waste handlers who suffered a sharp injury, 10 (19.2%) were infected with HCV virus, while 223 (97.4%) were free of the virus (Table 3).

**Table 3:** Risk factors and their association with HCV toward waste handlers in public hospitals in Sidama region, Ethiopia, 2022 (*n* = 282).

Variables	Response	Anti-HCV status		Pearson chi square	*P*-value
		Positive *n* (%)	Negative *n* (%)		
Family history of HCV infection	Yes	4 (3.1)	124 (96.9)	258.05	0.002*
	No	12 (8.3)	133 (91.7)		
Multiple sexual partners	Yes	12 (26.67)	33 (73.33)	140.12	0.042*
	No	4 (1.6)	232 (98.4)		
Sharp injury	Yes	10 (19.2)	42 (80.8)	135.78	0.037*
	No	6 (2.6)	223 (97.4)		
Taking technical training	Yes	3 (1.5)	192 (98.5)	145.74	0.001*
	No	9 (13.2)	59 (86.8)		
Using personal protective equipment	Yes	11 (5.1)	204 (94.9)	205.15	0.004*
	No	5 (10.2)	44 (89.8)		
Tattooing on body/gum	Yes	10 (12.5)	70 (87.5)	0.006	0.260
	No	6 (3.1)	189 (96.9)		
Contact with jaundiced patient without personal protective equipment	Yes	6 (2.5)	231 (97.5)	208.23	0.000*
	No	10 (22.7)	34 (77.3)		
Exposure to blood other body fluid splashes in the nose and eyes	Yes	7 (17.1)	34 (82.9)	254.74	0.000*
	No	9 (3.8)	231 (96.2)		
Unprotected sex	Yes	4 (8.5)	43 (91.5)	78.54	0.000*
	No	12(5.1)	222(94.9)		

* Significant variable.

The article "Generalized linear modeling of HCV infection among medical waste handlers in Sidama region, Ethiopia" was published in 2025. Journal: Front Epidemiol.

During waste collection, the majority of study participants (50%) wore gloves, followed by masks (41.8%), gowns (5%), and protective eyewear (3.2%). Among the 141 study participants who used gloves during waste collection, 121 (85.83%) were females and 20 (14.17%) were males, with no males (0%) wearing protective eyewear (Table 4).

**Table 4:** Use of personal protective equipment by sex among waste handlers in Sidama region, Ethiopia, 2022 (*n* = 282).

Personal protective equipment	Male (%)	Female (%)	Total (%)
Gloves	20 (14.17)	121 (85.83)	141 (50)
Masks	6 (5.1)	112 (94.9)	118 (41.8)
Protective eyewear	0 (0)	9 (100)	9 (3.2)
Gowns	10 (71.4)	4 (28.6)	14 (5)

### Waste handling practices

According to this research, only 97 (34.4%) of participants took part in an infection prevention or universal precaution training program. About 141 (50%) reported taking immediate action following blood exposure accidents (soap washing, disinfection). 114 (40.4%) of the study participants reported changing their gloves on a regular basis during waste collection for personal protection. On the other hand, more than half of the study participants 200 (70.9%) have a history of exposure to any form of bodily fluid, such as waste contaminated by body fluids (blood, peritoneal, pericardial, pleural, and so on). About 221 (78.4%) of the study participants reported a history of needle stick injury. The practices of waste handlers to prevent different infections and their association with HCV infection are shown in Table 4. As indicated, odds of begin infected by HCV for waste handlers who did not face needle stick injury were 0.58 times (OR = 0.58. 95% CI = 0.23–0.96, *P* = 0.000) lower than odds of being infected by HCV who faced needle stick injury during waste collection (Table 5).

**Table 5:** Association of practices to prevent infections and HCV infection status of among waste handlers (*n* = 282).

Variables	Response	*n* (%)	Anti-HCV status		Pearson chi square	OR (95%, CI)	*P*-value
			Positive *n* (%)	Negative *n* (%)			
Do you always change gloves during waste collection?	Yes	114 (40.4)	7 (43.8)	107 (40.4)	0.048	1	0.892
	No	167 (59.2)	9 (56.2)	158 (59.6)		0.89 (0.56–8.17)	
Have you ever faced needle stick injury?	Yes	221 (78.4)	9 (64.28)	60 (22.6)	85.69	1	0.000*
	No	60 (21.3)	5 (35.71)	205 (77.4)		0.58 (0.23–0.96)	
Have you ever exposed to any types of body fluids?	Yes	200 (70.9)	0 (0)	80 (30.2)	156.5	1	0.002*
	No	81 (28.7)	16 (100)	185 (69.8)		0.145 (0.05 –0.82)	
Do you take immediate action after blood exposure accidents (soap washing, disinfection)	Yes	141 (50)	13 (81.2)	138 (54.3)	278.15	1	0.004*
	No	129 (45.8)	3 (18.8)	116 (45.7)		2.156 (1.14 –6.26)	
Do you participated in training program about infection prevention	Yes	97 (34.4)	16 (13.6)	81 (49.4)	246.5	1	0.000*
	No	185 (65.6)	102 (86.4)	83 (50.6)		3.254 (2.15–5.87)	

* Significant variable.

The article "Generalized linear modeling of HCV infection among medical waste handlers in Sidama region, Ethiopia" was published in 2025. Journal: Front Epidemiol.

### Assessing model fit

The overall significance is tested, which is derived from the likelihood of observing the actual data under the assumption that the model that has been fitted is accurate. The deviance is the log-likelihood of the final model to the loglikelihood of a null model with no predictor variables. The deviance between −2*log-likelihood for the final model is 7,849.34 and for the null model is 13,508.64. Therefore, the full model gets smaller deviance, which is a good fit to the dataset.

In an effort to identify which model may be better used to model the data, values of AIC and BIC were also computed and displayed in Table 6. As indicated, AIC and BIC values decrease as we move from the null model (intercept only model) to the full model. This provides a rough indicator that the model fit improves as we add the independent variables. Finally, the information measures confirm that the full model fits the data much better than the null model. Therefore, the full model provided a good fit to the data.

**Table 6:** Comparison of null and full models using deviance, AIC, and BIC.

Selection criteria	Null model	Full model
Deviance	13,508.64	7,849.34
AIC	9.36	4.30
BIC	−4,061.91	−10,576.67

### Factors associated with HCV infection among the waste handlers

Exposure to blood, multiple sexual partners, sharp injury, taking technical training, not using personal protective equipment, contact with jaundiced patient, family history of HCV infection, unprotected sex were included into the model as these variables had *P*-value less than 0.05 in bivariate analysis (Table 7). Among a total of 282 waste handlers, 16 (5.7%) (95% CI = 4.2–8.7) were infected with HCV. HCV infection was 2 times more common among those waste handlers who experienced sharp injury (OR = 2.77, 95% CI = 2.327–3.173, *P* = 0.036), when compared to those who were not injured with sharp materials, and odds of HCV infection among those waste handlers who used personal protective equipment during waste collection were 0.77 times less common (OR = 0.77, 95% CI = 0.032–0.937, *P* = 0.001), compared with those who did not use personal protective equipment. The odds of having HCV infection were 11.91 times and 3.65 times more common among waste handlers who had unprotected sex (OR = 11.91, 95% CI = 5.847–16.854, *P* = 0.001) and among those who had contact with jaundiced patient (OR = 3.65, 95% CI = 1.093–4.368, *P* = 0.005), compared with those who did not have multiple sexual partners and did not have contact with jaundiced patients, respectively (Table 7).

The article "Generalized linear modeling of HCV infection among medical waste handlers in Sidama region, Ethiopia" was published in 2025. Journal: Front Epidemiol.

**Table 7:** Analysis results of the final GLM.

Risk factor	Estimates	Std. Err.	*Z*	OR	*P* > |*Z*|	95% CI
Exposure to blood	2.112	0.511	4.13	8.26	0.037*	1.878–10.925
Multiple sexual partners	1.289	0.350	3.68	3.63	0.001*	2.751–5.808
Sharp injury	1.018	0.382	2.66	2.77	0.036*	2.327–3.173
Taking technical training	0.034	0.013	2.57	1.03	0.471	0.897–1.941
Not using personal protective equipment	−0.24	0.010	0.29	0.77	0.001*	0.032–0.937
Contact with jaundiced patient	1.294	0.054	23.80	3.65	0.005*	1.093–4.368
Family history of HCV infection	0.068	0.057	1.18	1.07	0.284	0.955–1.179
Unprotected sex	2.477	0.052	47.28	11.91	0.001*	5.847–16.854

* Significant variable.

## Discussion

Waste handlers are among high risk groups for infectious diseases like HCV. Estimates of HCV infection among waste handlers are required to determine the disease burden and, hence, develop preventative interventions. However, there are no data on the prevalence of HCV infection in this risk group in Sidama region, Ethiopia. Hence, this study provided HCV infection data and risk factors among waste handlers.

In this study, the prevalence of anti-HCV in waste handlers was high (5.7%). The prevalence we report appeared to be higher as compared with other similar studies in South Omo Zone, Southern Ethiopia (1.9%) (11), Northwest Ethiopia (1.13%) (12), Dire Dawa (0.96%) (13), and Bahir Dar (2.5%) (14). Although direct comparison is difficult, our finding appeared to be lower as compared to the prevalence reported among pregnant women attending antenatal care (ANC) in Western Ethiopia (8.1% anti-HCV) (15). The prevalence we report was almost similar with a pooled prevalence of HCV among healthcare workers in Africa (5.58%) (16), and it was much higher than the prevalence among healthcare workers in Jimma, Southwest Ethiopia (0.42%) (17) and Nekemte, Western Oromia (0.64%) (18). These disparities in prevalence could be attributed to population differences, sample size, study design, and diagnostic tools used.

A study conducted in Brazil showed that the prevalence among residential waste handlers was 4.3%, which was lower than what we found (19). Differences may be related to location, sample size, level of knowledge and attitude, and commitment to prevention and control. Although direct comparison is difficult due to methodological and study population differences, the prevalence we reported appeared to be higher than a previous estimate of HCV infection among mothers in Jijiga, Eastern Ethiopia (20), prisoners in Jimma Town, Southwest Ethiopia (21), pregnant women in southern Ethiopia (22), voluntary blood donors in Wolaita, South Ethiopia (23), volunteer blood donors in Arba Minch SNNPR, Ethiopia (24) and among diabetic patients in Debre Tabor, Northwest Ethiopia (25). The prevalence we report was higher as compared with the studies in Jimma, South West Ethiopia (26) and Iran (9.5%) (27). These disparities may not be surprising given that some of the studies were not from the same risk group and some were done with the detection of both hepatitis C virus RNA and anti-HCV antibody, whereas our study only detected anti-HCV antibodies. The study implies that waste handlers' infection control and safety methods could be improved. To limit the risk of HCV exposure, reinforce the necessity of wearing personal protective equipment and adhering to strict hygiene practices.

The article "Generalized linear modeling of HCV infection among medical waste handlers in Sidama region, Ethiopia" was published in 2025. Journal: Front Epidemiol.

Anti-HCV prevalence was higher in the age group greater than or equal to 37 years than in the age group less than 37 years, although the difference was not statistically significant. Several studies revealed similar findings (28, 29). This increase in the rate of anti-HCV positivity with age could be attributed to the increased risk of HCV infection with time. The study recommends that targeted screening programs for older age groups, enhancing infection prevention methods, and maintaining education on HCV transmission hazards for all age groups, especially older workers, are important. Female waste handlers had higher anti-HCV positivity than male waste handlers, although this difference was not statistically significant (*P* = 0.132). This discrepancy may be attributed to the fact that the majority of respondents (87.2%) were females, which could be the source of the disparities. Married waste handlers were 2.051 times more prone to be infected by HCV than unmarried waste handlers, and the difference was not statistically significant (*P* = 0.295). Some of our findings were corroborated by results reported from Yemen, including 5.41% HCV infection in married and 4.35% in single waste collectors, which were not statistically significant (30). Our study recommend that additional research into the living conditions, household habits, or shared risk behaviors could offer insights into why married waste handlers may show higher, though not significant, rates of HCV infection. HCV infection was significantly lower among waste handlers with secondary or higher educational status compared to waste handlers with elementary or lower education levels (*P* = 0.000). Another study has validated this finding, with a higher frequency of HCV in people with primary education than in other categories (31). Offering targeted health education programs for waste handlers with lower education levels may help lessen the risk of HCV transmission.

The article "Generalized linear modeling of HCV infection among medical waste handlers in Sidama region, Ethiopia" was published in 2025. Journal: Front Epidemiol.

In this study, more than half of waste handlers had received technical training about infectious waste management, which did not show any statistical association with HCV infection. This is consistent with the result of study conducted in Dire Dawa (13). Protective measures such as extensive training and supervision for waste handlers on appropriate utilization of personal protective equipment such as gowns, gloves, masks, boots, and eye protection may reduce the incidence of sharp injuries and splash exposures. However, among this key worker group, only 141 (50%) of them used disposable gloves, 118 (41.8%) face masks, 9 (3.2%) protective eyewear, and 14 (5%) gowns. This result is consistent with other studies (32, 33). Our research revealed that no male waste handlers (0%) used protective eyewear. In similar investigations conducted in Jeddah, Saudi Arabia (34) and Dhaka, Bangladesh (35), 0% of male waste handlers wore protective eyewear. This indicates inadequate utilization of personal protective equipment and highlights the need to strengthen training and supervision.

In our study, exposure to sharp injury in the workplace accounts for 19.2% of infection with HCV, which is inconsistent with the WHO estimate that exposure to sharps in the workplace accounts for 40% infection with HCV. This variation may be due to sample size difference. The present study showed that 18.6% of waste handlers had sharp injuries while handling waste. This finding was higher than findings among the waste handlers at tertiary care hospitals of Karachi (36). The present study found 3.1% positive HCV infection rate among waste handlers with a family history of HCV infection. A higher result was obtained in Yemen (30), which reported a 5.66% positive rate among those with a family history of hepatitis C. This variation could be attributed to differences in healthcare infrastructure, access to treatment, and public health policies, and the study recommended expanding screening programs for family members of HCV-infected individuals, particularly those who work in high-risk occupations such as waste disposal. Taking technical training, tattooing on body/gum and family history of HCV infection demonstrated statistical associations in different research conducted in southern Ethiopia (37) whereas these variables did not show any association with the infection rates of HCV among our study participants. Our study suggested that exposure to blood, multiple sexual partners, sharp injury, not using personal protective equipment, contact with jaundiced patient, and unprotected sex were a possible pathway for HCV transmission among waste handlers. Some of these findings corroborated the study from northeast Ethiopia (38). The present study showed that HCV infection was 8 times more common among waste handlers who were exposed to blood (*P* = 0.037), when compared to those not exposed to blood, and the odds of having HCV infection were 3.63 times (*P* = 0.001) more common among waste handlers who had multiple sexual partners than those who did not have multiple sexual partners, which were statistically significant. These findings were supported by studies conducted in Spain (39), North West Ethiopia (40), Slovakia (41). Our study recommended that waste handlers strictly adhere to safety rules to avoid direct contact with blood, and that educational programs emphasizing the need of safe sex be adopted.

The article "Generalized linear modeling of HCV infection among medical waste handlers in Sidama region, Ethiopia" was published in 2025. Journal: Front Epidemiol.

Although the study conducted on the same study subjects in Sidama, Ethiopia showed that waste handlers had optimal level of knowledge, attitude and practice on several aspects of HCV (10), the prevalence of HCV among the same group was high (5.7%). This controversy may be due to the fact that the rules in the hospitals about color-coding segregation of wastes and commitments of waste handlers to use personal protective equipment may be very weak.

### Strength and limitation of the study

This study's extensive scope, which encompasses a wide range of healthcare facilities and geographical locations, may improve the findings' representativeness. However, we recognized certain limitations. The study was conducted in randomly selected hospitals in Sidama region, which may have recall bias, and screening for HCV was not conducted during employment and this made it difficult to identify whether the observed infection was before or after employment as waste handlers. Confirmatory test, like ELISA (Enzyme-Linked Immunosorbent Assay), was not used due to a shortage of laboratory equipment.

## Conclusion

The infection of HCV among waste handlers in public health hospitals in Sidama region, Ethiopia was higher compared to other findings. The high prevalence identified in this study indicated a strong need to scale up preventive efforts and strategic policy directions to limit the spread of this virus in the study area. The study recommended that hospitals should create awareness and work-related exposure prevention should be the first plan to reduce the risk of HCV infection among waste handlers. The significant demographic variable that was correlated with HCV infection was educational level of waste handlers. Adoption of more safe ways for waste collection and extensive training and supervision about appropriate use of personal protective equipment should be considered to reduce the infection of HCV.

The article "Generalized linear modeling of HCV infection among medical waste handlers in Sidama region, Ethiopia" was published in 2025. Journal: Front Epidemiol.

## Data Availability

The original contributions presented in the study are included in the article/Supplementary Material, further inquiries can be directed to the corresponding author.
